RETRACTED

# Analysis of Privacy-Preserving Edge Computing and Internet of Things Models in Healthcare Domain

**DOI:** 10.1155/2021/6834800

**Published:** 2021-12-30

**Authors:** Naif Almusallam, Abdulatif Alabdulatif, Fawaz Alarfaj

**Affiliations:** ^1^Department of Computer Science and Information, Imam Mohammad Ibn Saud Islamic University (IMSIU), Riyadh, Saudi Arabia; ^2^Department of Computer Science, College of Computer, Qassim University, Buraydah 51452, Saudi Arabia

## Abstract

The healthcare sector is rapidly being transformed to one that operates in new computing environments. With researchers increasingly committed to finding and expanding healthcare solutions to include the Internet of Things (IoT) and edge computing, there is a need to monitor more closely than ever the data being collected, shared, processed, and stored. The advent of cloud, IoT, and edge computing paradigms poses huge risks towards the privacy of data, especially, in the healthcare environment. However, there is a lack of comprehensive research focused on seeking efficient and effective solutions that ensure data privacy in the healthcare domain. The data being collected and processed by healthcare applications is sensitive, and its manipulation by malicious actors can have catastrophic repercussions. This paper discusses the current landscape of privacy-preservation solutions in IoT and edge healthcare applications. It describes the common techniques adopted by researchers to integrate privacy in their healthcare solutions. Furthermore, the paper discusses the limitations of these solutions in terms of their technical complexity, effectiveness, and sustainability. The paper closes with a summary and discussion of the challenges of safeguarding privacy in IoT and edge healthcare solutions which need to be resolved for future applications.

## 1. Introduction

Recent years have seen an incredible revolution in the healthcare industry. The Internet of Things (IoT) has added an altogether other dimension to healthcare technology. The IoT promotes sustainability in the healthcare industry by effectively facilitating patient treatment and minimizing the impact of the disease or preventing it entirely [1].  Figure 1 shows an overview of edge computing and Internet of Things paradigms. Edge computing paradigm takes place closer to the physical IoT units (e.g., a user or the data source) which in turns plays a critical role as a midpoint to lower latency and saves bandwidth to the cloud.

The IoT has created applications barely thought possible, such as Remote Patient Monitoring (RPM) via wearable devices, embedded devices (e.g., pacemakers and infusion pump) and health monitoring devices for general consumer market [2]. The IoT ecosystem in healthcare is not limited to these medical devices alone. It encompasses sensors and all those devices which are powered by the Internet and collects and communicates the data to provide time-dependent critical services to different actors involved in a particular healthcare system setting [3, 4]. However, regardless of the versatility of the IoT, 41.4 million EHRs (Electronic Health Records) were compromised by data breaches in 2019 alone [5]. The trend continued with multiple data breaches reported in 2020, especially during COVID-19. A study conducted in 2020 confirmed that 90% of communications occurring via IoT devices are unencrypted, making data more vulnerable to unauthorized exposure [6]. These data breaches compromise the privacy of users with regard to their Personal Identifiable Information (PII) and location, which can have serious consequences [7]. Various privacy-preservation techniques have been devised by researchers for implementation within healthcare solutions. However, the success of these techniques is totally dependent on the way they are implemented and on the characteristics of underlying infrastructure, i.e., on the strengths and weaknesses of the IoT and edge computing environments. The computation power of IoT devices is not on par with cloud computing facilities, making cloud services and alike essential for IoT. The long-distance data in transit which is communicated to the cloud server is vulnerable to all kinds of cyber-attacks which can breach the privacy and confidentiality of data and users. The data which comes under the umbrella of HIoT (Healthcare Internet of Things) or IoMT (Internet of Medical Things) is susceptible to such attacks because it is highly sensitive and represents higher stakes for both patients and care givers [3, 8].

RETRACTED

As a means of addressing the high latency and privacy issues of cloud computing environments in the context of the IoT paradigm, edge computing offers significant prospects. Edge computing enables computation to take place close to IoT devices, rendering the data in real time and reducing the potential risk of data leakage during transit [7, 9, 10]. Although the latency issue is handled by the edge infrastructure, the cloud can still provide nondynamic analytics and AI functionality for huge data collected to provide substantial services for IoT and edge end-devices [11–13]. Nevertheless, the nature of edge services demands an unconventional set of security and privacy-preserving mechanisms. These must be in accordance with its characteristics (i.e., lightweight, efficient, and resource-constrained and distributed multiple sources of incoming data) [12, 14].

Both the IoT and edge computing offer sophisticated services that can shape and improve the modern healthcare sector; however, their distributed nature needs to be kept in check in order to ensure the privacy of users' data including the user patterns, identity, and location [7]. The risk of data exposure is not only due to data leakage from faulty devices or hacker attacks. Service and infrastructure providers can also pose enormous risks to data security. Personnel can use the data for personal gain, sell the data to other third parties, or constitute an insider threat from the provider's own organization [15, 16]. Similarly, government agencies can use the location data of users to monitor the spread of COVID-19 in the current pandemic; however, the PII collected must not be publicly accessible [6]. In this paper, the current situation regarding privacy preservation in the IoT and edge solutions for the healthcare ecosystem is analyzed and discussed.

This paper is organized as follows.  Section 1 introduces the focus of this study.  Section 2 of the paper provides a survey of the present literature on the privacy concerns associated with edge computing and IoT healthcare solutions. Sections 3 and 4 describe the privacy mechanisms used in edge computing and IoT healthcare solutions, including their strengths and weaknesses.  Section 5 discusses the gaps found in the current privacy-preserving solutions, and Section 6 concludes the paper and suggests future research paths.

## 2. Literature Survey

Numerous research articles of existing literature were found that demonstrated the use of edge computing and the IoT in the healthcare industry. However, interestingly, less research has been conducted on privacy preservation in computing paradigms with regard to the healthcare industry. This section summarizes the current techniques used in edge and IoT applications to ensure data privacy in the healthcare domain. The authors of [17] proposed a lightweight and privacy-preserving fog-assisted information sharing scheme for healthcare data based on a hierarchical attribute-based encryption. Furthermore, Giri et al. proposed a security protocol called SecHealth to secure healthcare sensor data transmission to a fog-based servers [18]. Al Hamid et al. proposed a privacy-privacy model for big data in a healthcare domain by using edge computing paradigm with pairing-based cryptography [19]. Anajemba et al. developed an efficient sequential convex estimation optimization algorithm to improve physical layer security [20]. The authors in [21] demonstrate an IoT system which makes use of an encryption scheme to resist attacks by using quantum level computations, i.e., SIMD (Single Instruction Multiple Data) and SHE (Somewhat Homomorphic Encryption). The system collects images of patients' retinas, processes them via a cloud service, and returns the results to the practitioners. After carefully analyzing the results, practitioners make a diagnosis and send it back to the cloud service and the patients. The encryption used at every stage ensures data confidentiality and patient privacy.

RETRACTED

Similarly, a systematic review conducted in [15] investigated the available IoT-based health sensors and lists the security and privacy issues related to health data collected by these sensors. They discuss how to tackle those privacy issues at different stages of data processing using various techniques such as hashing, encryption, involving Trusted Third Parties (TTP), and anonymization schemes. Many researchers have used complete or partial blockchain technology to safeguard the privacy and integrity of data obtained from IoT devices. [4] have treated Electronic Health Records (EHRs) as blockchain transactions, each having a unique identifier and a hashed value. The unique identifier is encrypted with their proposed encryption scheme which is devoid of a decryption key. The encryption is dependent on the 32-bit random number generation, negative-AND, and modulus operations.

The issue of user privacy is predominant in wearable devices as they are usually programmed to broadcast the data, mostly using low frequency devices like BLE or Bluetooth. The authors of [22] have proposed an IoT architecture which ascertains the provenance of the data and dictates a device subscription policy. The devices that are to communicate undergo a meta data encryption. The devices which are subscribed can only receive the data and have decryption keys. Further evaluations are made to check the resilience and effectiveness of the architecture. The use of lightweight homomorphic encryption and anonymization techniques such as differential privacy (DP) is also evident in edge computing solutions, as shown in [23–25]. The researchers in [26] have made use of hardware-based solutions such as Intel's Software Guard Extension (SGX) implementation and blockchain, applying these simultaneously to prevent the exposure of sensitive data. The combination of blockchain technology and InterPlanetary File Systems (IPFS) has been proposed by the authors of [27] to ensure the privacy of data in transit and storage within a decentralized environment in IoMT. Data hiding (DH) mechanisms, specifically the Pixel Repetition Method (PRM) in steganography, has been combined with encryption schemes by the researchers in [5] to test a framework which can prevent and detect a privacy breach. The aim of the framework is to utilize the edge nodes to perform the computations on medical images in real time.

RETRACTED

The next sections will examine other healthcare solutions and highlight the challenges associated with the safeguarding of privacy in the domains of edge computing and IoT.

## 3. Privacy Preservation IoT based Healthcare Solutions

The IoT devices with their constrained resources are not enough to compute traditional cryptographic keys [29]. Hence, this eliminates the possibility of conventional cryptography mechanisms alone being used by IoT devices. Their limited resources led to the consolidation of edge and other computing paradigms in the healthcare industry. For example, in [28], the authors proposed a privacy-preserving strategy to eliminate the risk of data leakage during the data handling process. However, they had to introduce a third-party cloud platform to handle the computations involved in encryption schemes. Various anonymization schemes have been devised for use within healthcare sensor networks as in [30] who proposed a health data anonymization algorithm including an encryption scheme to ensure the privacy of sensitive data. It can be a valid solution but cannot be an optimal or an efficient one considering the bandwidth required, computation, cost, and latency involved. Apart from lacking computational power, the IoT devices have other limitations including low memory, being in low power mode for longer usage, low connectivity rate, and a frequently-changing context due to mobility [31]. Surveys on the issue of IoT healthcare security and privacy found that authorization and impersonation were the leading causes of data leakage [34, 35]. Hence, there is a focus on authentication- and authorization-based, privacy-preservation solutions for IoT healthcare systems. For example, a secure-anonymous biometric-based user authentication scheme (SAB-UAS) is proposed in [33], eliminating the risk of sensitive data exposure through unauthorized access. The authors themselves suggest the improvements required for the SAB-UAS protocol in terms of latency, routing overhead, and overall network performance. Information linkage is another threat discussed in academia in regard to heterogeneous IoT systems, specifically wearables and hand-held devices, etc., which might share sensitive health data with irrelevant services [36].

Pseudonymization and anonymization techniques are used as an added security layer in a health IoT application to eliminate the possibility of identifying an individual after a data breach [32]. In this scenario, aside from the technical aspects, the legal framework is also required to handle the concerns of all stakeholders involved.  Table 1 lists the main privacy-preservation solutions in healthcare IoT along with the limitations that need to be addressed.

RETRACTED

## 4. Privacy Preservation Edge Computing-Based Healthcare Solutions

The implementation of noninvasive and privacy-preserving solutions using edge computing is technically more feasible. Because edge devices have more computing power than IoT devices, the chances of successfully incorporating compute-intensive security and privacy methods are increased. However, compute-intensive solutions incur greater overheads. Research is being conducted to develop cost-effective privacy-preserving mechanisms. For example, in [14], a Lightweight Privacy-Preserving Data Aggregation Scheme for Edge Computing (LDPA-EC) has been proven to reduce the computational overheads while maintaining the privacy and integrity of data. The private data of patients/users which are collected by wearable devices are accessed by edge nodes for further calculations. If the edge nodes are compromised, it becomes a challenging task to prevent the data from being accessed by those nodes [26]. To tackle this issue, different encryption schemes are consolidated to make data secure within edge nodes. The encryption schemes include identity-based, attribute-based, proxy re-encryption, and homomorphic encryption [7, 25, 37]. Blockchain technology is a trending candidate in edge solutions to privacy issues [38]. As the data which is collected by IoT devices is a one-time venture and cannot be modified once collected, the storage of these one-time collections as blockchain transactions is an effective privacy-preserving solution [13].

Most of the research on privacy-preserving solutions in edge computing focuses on devices. However, in [11], authors discuss user-centric edge solutions where it is assumed that a user's lack of awareness can pose a risk to his/her private information. In this scenario, virtualization, particularly making use of network function virtualization (NFV) [11] to group services like firewalls, content inspection, authorization, and authentication for individual users, can reduce the risk significantly. The heterogeneous nature of private data aggregation in edge device/server and its sharing of the resources among numerous devices and services within a network poses a great risk of data exposure and loss [38].  Table 2 lists the prevalent privacy-preserving solutions in healthcare edge computing, along with the limitations that need to be addressed.

## 5. Discussion

It is evident from above stated segments of the research that not a single computing paradigm can sufficiently handle privacy-preserving mechanisms on its own for healthcare solutions. Therefore, for an effective privacy preservation, the consolidation of computing paradigms is necessary.  Table 3 summarizes the challenges associated with the privacy-preservation solutions offered by edge and IoT technologies. A combination of IoT and edge computing not only provides efficient dynamic services to the consumers but can also create consumer trust by maintaining their privacy.

RETRACTED

Moreover, by analyzing the aforementioned solutions, it can be concluded that the more decentralized the design of a healthcare solution, the more it can prevent the leakage of private data. But where decentralization prevents a single point of failure and is a benefactor for differential privacy mechanism, it also introduces intricate complexity in overall system performance. Heterogeneity and the decentralized nature of edge computing also make it more difficult to achieve effective and secure scale-up of services. Although the new 5G wireless standard is enabling more device-to-device interaction, the communication protocols are vulnerable to cyber-attacks aimed at accessing information about the type of IoT device and its configuration [39]. Furthermore, this vulnerability can be exploited to gain access to sensitive biological information from e-health solutions and devise a cyber-physical attack against a user. Hence, not only should privacy-preservation modules be included in the IoT environment but hardware and protocols should be given priority as well.

Apart from the technological aspects of privacy-preserving solutions in computing paradigms, the willingness to share the data by users should also be considered. The healthcare solutions proposed by developers and service providers should be carefully considered so that only necessary information is being collected, not an excessive amount of data. By adhering to the Keeping Privacy by Design (PbD) [32] principles from the outset, developers could provide solutions that minimize the number of potential risks. Currently, there is a lack of trust layers or trusted management systems for resource exchanges between IoT devices, edge devices, and cloud servers [37]. The formulation of clear privacy policies for data collection, handling, and transmission could also help to safeguard data privacy preservation and streamline investigation in the event of any breach.

## 6. Conclusion

This paper has discussed the importance of privacy preservation, especially in the healthcare sector where it is critical to ensure the privacy of patients' data. The paper outlined and discussed privacy preservation solutions in IoT and edge environments. Furthermore, it identified the limitations of each one of these computing paradigms when it comes to securing and handling private data. It can be concluded that the interdependence of computing paradigms adds some complexity to solutions but is nevertheless essential as a means of providing effective privacy-preserving mechanisms. In the near future, the widespread adoption of 5G will add robustness to privacy preservation computations although it may introduce new challenges. The secure interoperability of IoT and edge end devices in different contexts is a vast area of research meriting in-depth investigation.

RETRACTED

## Figures and Tables

**Figure 1:** An overview of edge computing and Internet of Things paradigms. Edge computing paradigm takes place closer to the physical IoT units (e.g., a user or the data source) which in turn plays a critical role as a midpoint to lower latency and saves bandwidth to the cloud.

**Table 1:** Privacy-preserving solutions in IoT-based healthcare and the associated challenges.

Privacy-preserving IoT-based healthcare solutions	References	Challenges
Quantum level computations SIMD-SHE	[21]	Dependence on other platforms (cloud computing)
Complete or partial use of blockchain	[4]	Need excessive computation resources
Data encryption schemes	[15, 22]	Low computation resources and high latency
Cryptography mechanisms	[15, 28] [29]	Limited resources
Data pseudonymization and anonymization schemes	[30–32]	Low bandwidth and network performance, absence of legal framework
Secure authentication scheme (SAB-UAS)	[33]	Low latency and network performance with high cost

**Table 2:** Privacy-preserving solutions in edge computing-based healthcare and the associated challenges.

Privacy-preserving edge computing based healthcare solutions	References	Challenges
Anonymization techniques such as differential privacy	[23, 24]	Complexity due to decentralization
Hardware level solution (SGX)	[26]	High cost
Blockchain technology	[13, 38] [26, 27]	Complex decentralization and high overheads
Data hiding mechanism (PRM)	[5]	Intercommunication complexity
Encryption schemes	[7, 14, 25] [5, 37]	High cost
Network function virtualization (NFV)	[11]	Complexity introduced by heterogeneity

**Table 3:** Summary of privacy preservation challenges in both IoT and edge computing-based healthcare solutions.

Privacy preservation challenges computing	IoT	Edge
(1) Less computing power for executing privacy solutions.	✓	
(2) Inefficient performance for real time secure processing.	✓	
(3) Limited resources with regard to bandwidth.	✓	
(4) Lack of privacy policies.	✓	✓
(5) Absence of trust management layers between computing paradigms.	✓	✓
(6) Lack of user awareness about sharing their own data.	✓	✓
(7) Limited resources with regard to memory.	✓	✓
(8) High mobility of devices introduces the challenge to keep the privacy preservation mechanisms intelligent and dynamic.	✓	✓
(9) Dependence on other platforms for optimal performance.	✓	
(10) Heterogeneous nature impels for complex intercommunication between devices and among platforms.	✓	✓
(11) Decentralized architecture's complexity.		✓
(12) Requirement of unconventional lightweight privacy mechanisms.		✓
(13) Compatibility issues within devices can lead to misconfiguration and thus data exposure.		✓
(14) High computational overheads.		✓
(15) Possibility of hardware (device/node) compromise.	✓	✓

RETRACTED

## Data Availability

No data were used to support this research.
